The article "The significance of the change pattern of serum CA125 level for judging prognosis and diagnosing recurrences of epithelial ovarian cancer" was retracted in 2022. Reasons: original data or images not available; lack of ethics approval or compliance; missing or withdrawn patient consent.

# The significance of the change pattern of serum CA125 level for judging prognosis and diagnosing recurrences of epithelial ovarian cancer

**DOI:** 10.1186/s13048-016-0266-3

**Published:** 2016-09-15

**Authors:** Zhi-jun Yang, Bing-bing Zhao, Li Li

**Affiliations:** Department of Gynecologic Oncology, Affiliated Tumor Hospital of Guangxi Medical University, 71# Hedi Road, Nanning, Guangxi 530021 People’s Republic of China

**Keywords:** CA125, Change pattern, EOC, Prognosis, Recurrence

## Abstract

**Background:**

Ovarian cancer has the highest mortality rate of the three main malignant tumors of the female reproductive system, with a 5-year overall survival (OS) of only 20–30 %. Approximately 70 % of patients relapse without being cured. To explore the significance of serum CA125 level pre-treatment and the change pattern of CA125 post-treatment for judging prognosis and diagnosing recurrences of epithelial ovarian cancer (EOC).

**Methods:**

A radioimmunoassay was used to continuously monitor levels of serum CA125 in 152 patients with EOC. The first test was done before surgery, then once a month after surgery for more than two consecutive years. The data were analyzed by using Kaplan-Meier curves and the log-rank test, stratified chi-square test, Pearson correlation analysis, and multivariate Cox regression analysis.

**Results:**

(1) There was a relationship between patient outcomes and the serum CA125 levels before treatment and the extent and speed of serum CA125 decrease after treatment. The outcomes of patients with pre-treatment serum CA125 ≤ 35 U/ml were better than those with serum CA125 > 35 U/ml; the outcomes of patients with serum CA125 who had a logarithmic decrease or a decrease to normal within a month after treatment were also better than those with a non-logarithmic decrease or a decrease to normal that took longer than a month. (2) The results of multivariate Cox regression analysis showed that serum CA125 levels before treatment and a decreased speed of decline after treatment were independent prognostic factors; (3) The mean level of serum CA125 at relapse was 116.28 U/ml. The average time from serum CA125 increase to detection of a recurrent lesion by physical or imaging examination was 122 days. The correlation coefficient of serum CA125 level increase and tumor recurrence time was −0.674. (4) The area under the Receiver Operating Characteristic (ROC) curve of serum CA125 for diagnosing EOC recurrence was 0.879, and the sensitivity and specificity were 67.39 and 86.79 %, respectively.

**Conclusions:**

It is important to monitor serum CA125 levels pre-treatment and the change pattern of CA125 post-treatment for judging prognosis and diagnosing recurrences of EOC.

The article "The significance of the change pattern of serum CA125 level for judging prognosis and diagnosing recurrences of epithelial ovarian cancer" was retracted in 2022. Reasons: original data or images not available; lack of ethics approval or compliance; missing or withdrawn patient consent.

## Background

Ovarian cancer has the highest mortality rate of the three main malignant tumors of the female reproductive system, with a 5-year OS of only 20–30 % [1]. The early stages of ovarian cancer have no overt or classical clinical symptoms and most patients are diagnosed in advanced stages, so clinical treatment and prognosis are not satisfactory. Approximately 70 % of patients relapse without being cured. Early diagnosis of recurrences of EOC has great significance for its treatment and prognosis. This article retrospectively evaluates the change pattern of serum CA125 level during the whole treatment process of EOC patients, analyzes the relationship between patient’s disease status and the level of serum CA125, and explores the significance of the change pattern of serum CA125 level for judging prognosis and diagnosing recurrences of EOC.

## Methods

### Clinical data of cases

#### Subjects

A total of 152 patients with ovarian cancer treated at our hospital from January 2005 to December 2011 were included in the study. Diagnoses of all patients were confirmed by histopathology. All patients were treated primarily with optimal cytoreductive surgery (hysterectomy, bilateral salpingo-oophorectomy, omentectomy, pelvic lymph node dissection, and para-aortic lymph node dissection at the level of the inferior mesenteric artery, and appendectomy for mucinous carcinoma) followed with platinum-based chemotherapy for 6 to 8 cycles. All patients had clinical complete remission after primary surgery and adjuvant chemotherapy and a disease free survival time of 6 months or more. The clinicopathological characteristics of patients were shown in Table 1.

**Table 1:** Clinicopathological characteristics of the patients

Pathology	
Histologic type(n)	152
Serous	104
Mucinous	31
Others(mixed,endometrioid,clear-cell carcinoma)	17
Median age (year)	46 (25–72)
FIGO stage(n)	152
I	53
II	30
III	69

### Follow up

All 152 patients were followed up to December 31, 2015. The median follow-up time was 82 months. At the end of the follow-up period, 117 patients were still alive. Among them, 46 patients had had relapses and 106 patients had not; all of the relapses were confirmed by histopathology.

### Peripheral serum collection and serum CA125 detection

Peripheral blood 2 ml was collected under written consent from the patients in the morning after fasting pre-treatment, post-treatment, during each chemotherapy, and at times of recurrence. The samples were stored at 4 °C for 2 h, centrifuged at 3000 rpm for 5 min, then the supernatant was collected and stored at −80 °C. A radioimmunoassay was used to detect the concentration of serum CA125, performed according to the manufacturer’s specifications; the normal value range is ≤ 35 U/ml.

The article "The significance of the change pattern of serum CA125 level for judging prognosis and diagnosing recurrences of epithelial ovarian cancer" was retracted in 2022. Reasons: original data or images not available; lack of ethics approval or compliance; missing or withdrawn patient consent.

### Statistical analysis

SPSS19.0 statistical software was used to analyze the data. Categorical data were analyzed by *χ*^2^ tests and continuous data were analyzed by rank-sum tests. The survival rate in different groups was analyzed by log-rank tests and stratification analyses were performed with stratified chi-square tests. Correlation analyses were performed using Pearson’s correlation test, and multivariate analyses were performed using Cox regression models. *P* < 0.05 was defined as statistically significant.

## Results

### The relationship between serum CA125 levels and progression-free survival (PFS) and OS

When patients with pre-treatment serum CA125 level ≤ 35 U/ml were compared with those with serum CA125 level > 35 U/ml, the median PFS was 52 and 36 months, respectively, *P* = 0.032, a statistically significant difference. The median OS of these 2 groups was 54 and 39 months, respectively, *P* = 0.023, a statistically significant difference (see Fig. 1).

**Fig. 1:** Relationship between levels of pre-treatment serum CA125 concentration and PFS, OS

Age, stage, and pathological types were used to perform a stratification analysis of each pre-treatment serum CA125 level, comparing the survival rate and calculating the odds ratio and 95 % confident interval distribution according to the results of the stratification analysis. As shown in Fig. 2, the survival rate in each serum CA125 level stratum has no significant difference by age, stage, or pathological type (*P* > 0.05).

**Fig. 2:** Odds ratio of survival rate and 95 % confidence distribution

### The relationship between prognosis and the extent and speed of serum CA125 decrease after treatment

When comparing patients with a post-treatment logarithmic decrease (shown as Fig. 3) of serum CA125 with patients without a non-logarithmic decrease, the median PFS was 45 and 34 months, respectively, *P* = 0.043, a statistically significant decrease. The median OS was 61 and 38 months, respectively, *P* = 0.038, a statistically significant decrease (see Fig. 4).

**Fig. 3:** Typical curve of CA125 logarithmic decrease

**Fig. 4:** Comparison of PFS, OS between different serum CA125 decrease patterns after treatment

We explored the relationship between patient outcome and the speed of serum CA125 decrease. Comparing patients in whom serum CA125 decreased to normal within a month with those that took more than a month, the median PFS was 45 and 38 months, respectively, *P* = 0.047, a statistically significant difference. The median OS was 56 and 38 months, respectively, *P* = 0.029, a statistically significant difference (see Fig. 5).

The article "The significance of the change pattern of serum CA125 level for judging prognosis and diagnosing recurrences of epithelial ovarian cancer" was retracted in 2022. Reasons: original data or images not available; lack of ethics approval or compliance; missing or withdrawn patient consent.

**Fig. 5:** Comparison of PFS, OS between different speeds of serum CA125 decrease after treatment

Multivariate Cox regression analysis was used to analyze the serum CA125 levels at pre-treatment, the extent and speed of serum CA125 decrease after treatment, and the increased level of serum CA125 in relapses. The results show that levels before treatment and decreased speed of decline of serum CA125 levels after treatment were independent factors (see Table 2).

**Table 2:** Cox regression analysis

Impact factor (CA125)	Partial regression coefficient	Relative risk	*P*
Levels before treatment	1.136	3.274	0.025
Decrease speed after treatment	2.164	6.213	0.002

### The relationship between serum CA125 levels (biochemical recurrence) and finding lesions by imaging examination

Fifty-one patients were diagnosed positive for a recurrence by imaging examination. Among them, 40 patients were true positive and 11 patients were false positive. Twenty-one patients (52.5 %) had serum CA125 ≥ 100 U/ml, 14 patients (35.0 %) had serum CA125 between 35–100 U/ml, and 5 patients (12.5 %) had serum CA125 ≤ 35 U/ml. Comparing patients with serum CA125 ≥ 100 U/ml with those with serum CA125 between 35–100 U/ml, *P* = 0.397, the difference was not statistically significant. Comparing patients with serum CA125 ≥ 100 U/ml with patients with serum CA125 ≤ 35U/ml, *P* = 0.003, the difference was statistically significant. Comparing patients with serum CA125 between 35–100 U/ml and those with serum CA125 ≥ 100 U/ml, *P* = 0.041, the difference was statistically significant. As we can see in Table 3, mainly patients with serum CA125 ≥ 100U/ml were diagnosed true positive by imaging examination and those diagnosed false positive by imaging examination were mainly patients with serum CA125 ≤ 35 U/ml.

**Table 3:** The relationship between serum CA125 levels in recurrences and finding lesions by imaging examinations

Serum CA125 levels after treatment (U/ml)	Imaging (CT, MRI) diagnosis		
	Positive (case %)	Negative (case %)	*P*
≥100^a, b^	21 (52.5 %)	2 (18.2 %)	0.397^a^
35–100^a, c^	14 (35.0 %)	3 (27.3 %)	0.003^b^
≤35^b, c^	5 (12.5 %)	6 (54.5 %)	0.041^c^
Total	40	11	

^a^: Comparison between patients with CA125 ≥ 100 U/ml and patients with CA125 35–100 U/ml

^b^: Comparison between patients with CA125 ≥ 100 U/ml and patients with CA125 ≤ 35 U/ml

^c^: Comparison between patients with CA125 35–100 U/ml and patients with CA125 ≤ 35 U/ml

Correlation analysis found that the average increased level of serum CA125 at relapse was 116.28 U/ml. The average time between serum CA125 level increase to finding a recurrent lesion by physical examination or imaging examination was 122 days. The correlation coefficient of serum CA125 level increases and tumor recurrence time was –0.674; i.e., the average increased levels of CA125 in relapsed patients and the average time of displaying recurrent lesions were negatively correlated. The higher the serum CA125 level was, the shorter the time before the recurrent lesion was detected (see Fig. 6).

The article "The significance of the change pattern of serum CA125 level for judging prognosis and diagnosing recurrences of epithelial ovarian cancer" was retracted in 2022. Reasons: original data or images not available; lack of ethics approval or compliance; missing or withdrawn patient consent.

**Fig. 6:** The scatter diagram of the average time of serum CA125 level increase to finding the recurrent lesion

### The significance of the change pattern of serum CA125 level post-treatment for diagnosing recurrence of EOC

In all of the patients, 35 U/ml was defined as the critical cutoff value for recurrence. Serum CA125 in 45 patients was > 35 U/ml, and among them 31 patients were diagnosed by pathology; in 107 patients, serum CA125 was ≤ 35 U/ml, and among them 15 patients were diagnosed by pathology. The area under the ROC curve was 0.879 for diagnosing an EOC recurrence by using serum CA125, and the diagnostic sensitivity and specificity was 67.39 and 86.79 %, respectively. The positive predictive value was 0.69, the negative predictive value was 0.86, the positive likelihood ratio was 5.10, and the negative likelihood was 0.38 (see Fig. 7).

**Fig. 7:** ROC of CA125 for diagnosing recurrences

## Discussion

### The significance of the change pattern of serum CA125 level post-treatment for judging recurrences of EOC

The clinical data statistical analysis shows that there was a relationship between patient outcomes and serum CA125 levels before treatment and the extent and speed of serum CA125 decrease after treatment. The outcomes of patients with pre-treatment serum CA125 ≤ 35 U/ml were better than those with serum CA125 > 35 U/ml. The outcomes of patients with serum CA125 logarithmic decrease or decrease to normal within a month after treatment were also better than those with a non-logarithmic decrease, or taking more than a month to decrease to normal.

Comparing patients with a serum CA125 logarithmic decrease and those with a non-logarithmic decrease, the median PFS was 45 and 34 months, respectively, *P* = 0.043, a statistically significant difference. Results of multivariate Cox regression analysis showed that CA125 levels before treatment and a decreased speed in decline of serum CA125 after treatment were independent prognostic factors.

The serum CA125 level pre-treatment is closely related to tumor size. The higher the serum CA125 levels, the larger the tumor lesions are, and the deeper and wider the tumor infiltrates, making cytoreductive surgery (CRS) harder. Whether CRS is successful or not has a great influence on continued treatment, so it affects prognosis. Eltabbakh et al. [2] explored influence factors of optimal CRS and found that 72 patients with advanced ovarian cancer could have an optimal CRS if serum CA125 was ≤ 500 U/ml. Vorgias et al. [3] analysed the relationship between the preoperative CA125 levels of 426 patients with Stage III/IV ovarian carcinoma and the surgical outcome. The data indicated preoperative CA125 is a good predictor for optimal CRS. The area under curve of the ROC curve was 0.89, 98 % C.I. = [0.828–0.952], indicating very good discriminating capability. The level of 500 IU/ml was found to have the most predictive power. The sensitivity of CA125 at that level was 78.5 %, the specificity 89.6 %, the positive predictive value 84.2 %, the negative predictive value 85.4 % and its accuracy 85 %. Furthermore, the likelihood ratio for correct discrimination between optimal and sub-optimal CRS, dropped sharply from 6.33, 95 % C.I. [5.19–10.91] at the level of 500 IU/ml to 0.58, 95 % C.I. [0.21–1.63] at the level of 600 IU/ml. The data indicate that the best threshold for this prediction proved to be 500 IU/ml. These patients may be candidates for neo-adjuvant chemotherapy treatment.

The article "The significance of the change pattern of serum CA125 level for judging prognosis and diagnosing recurrences of epithelial ovarian cancer" was retracted in 2022. Reasons: original data or images not available; lack of ethics approval or compliance; missing or withdrawn patient consent.

There is a close relationship between post-treatment serum CA125 levels and the size of residual lesions after CRS. The larger the residual size, the slower the serum CA125 level decreases. If the serum CA125 level does not decrease rapidly after CRS it always means that the residual lesions are large, the prognosis is worse, and the patients can relapse easily. The speed of serum CA125 decrease to normal after treatment has significance for diagnosing relapse to some degree. Patients with a high pre-treatment level of serum CA125 have a better prognosis if their serum CA125 decreases to normal rapidly after surgery, while patients with a low pre-treatment level of serum CA125 have a worse prognosis if their serum CA125 does not decrease to normal rapidly after surgery.

Systemic, regular, and full doses of chemotherapy are necessary, and after chemotherapy the serum CA125 levels decrease. The half-life of serum CA125 can show the changing rate of serum CA125 in early treatment by chemotherapy and we can judge the prognosis according to the half-life of serum CA125. Na et al. [4] showed that patients with a serum CA125 half-life of more than 20 days (group 1) have a 3.2 times greater risk of recurrence than those with a serum CA125 half-life of less than 20 days (group 2). The average relapse-free time of group 1 was 11 months and that of group 2 was 43 months. Digant et al. [5] Reported that reduction in CA125 after 3 months of therapy is associated with better overall survival in ovarian cancer. Patients without a significant decline in CA125 after 3 months of therapy have a particularly poor prognosis.

The article "The significance of the change pattern of serum CA125 level for judging prognosis and diagnosing recurrences of epithelial ovarian cancer" was retracted in 2022. Reasons: original data or images not available; lack of ethics approval or compliance; missing or withdrawn patient consent.

### The significance of the change pattern of serum CA125 levels post-treatment for diagnosing recurrence of EOC

Our data show that the serum CA125 level of most relapsed patients would rises. The average increased level is 116.28 U/ml; the average time between an increase in serum CA125 and detection of the recurrent lesion by physical examination or imaging examination is 122 days, and there is a relationship between the pattern of serum CA125 level increases and finding the recurrent lesion by physical or imaging examination. The increased level of serum CA125 has a negative correlation with the time before finding the recurrent lesion. The higher and faster serum CA125 increases, the shorter the time to find the recurrent lesion by physical or imaging examination. These results are similar to the results of Levy [6]. Levy’s team observed the change pattern of serum CA125 in relapsed patients with EOC and found that PFS or OS of relapsed patients with serum CA125 that increased slowly are longer than for those whose serum CA125 increased rapidly. In this study, the area under the ROC curve was 0.879, and the sensitivity and specificity for diagnosing recurrence were 67.39 and 86.79 %, respectively. The sensitivity of diagnosing recurrence was low, may be because of the following reasons: (1) The recurrent tumors are small and the levels of antigen may be too low to activate an antibody response. (2) There is a fibrous envelope around the cancer tissue which might block the release of the antigen into the blood circulation. (3) Chemotherapy drugs may have changed the biological behavior of the cancer cells. Some studies found that in patients with negative serum CA125, the negative rate of second surgical exploration was as high as 43.8 %. A previous study confirmed that serum CA125 is positive if the patients suffer from pelvic inflammation, endometriosis, pleura and peritoneum pathological changes, or liver cancer.

### Solutions for EOC patient with simple serum CA125 increases post-treatment

There is still a controversy about whether patients should receive treatment when their serum CA125 increases alone post-treatment [7, 8]. A prospective multicenter clinical trial showed that patient outcomes were not improved if chemotherapy was given when serum CA125 increased, and it reduced quality of life [9]. This may be because the tumor cells were not in the proliferation period and were not sensitive to chemotherapy drugs.

## Conclusions

CA125 is the most widely used tumor marker in ovarian cancer for diagnosis, monitoring disease and judging prognosis. Our study indicates that levels before treatment and decreased speed of decline of serum CA125 after treatment were independent factors. There is a negative correlation between pre-treatment CA125 level and prognosis, the sooner decrease of CA125 levels post-treatment the better prognosis are. When the serum CA125 levels after treatment increase over to 116.28 U/ml comprehensive examination would be used to identify whether recurrences occur. The average time from serum CA125 increase to detection of a recurrent lesion by physical or imaging examination was about 3 months. It is not recommend chemotherapy when patients serum CA125 increased alone after post-treatment. So It is important to monitor the change pattern of serum CA125 post-treatment for judging prognosis and diagnosing recurrences of EOC.

The article "The significance of the change pattern of serum CA125 level for judging prognosis and diagnosing recurrences of epithelial ovarian cancer" was retracted in 2022. Reasons: original data or images not available; lack of ethics approval or compliance; missing or withdrawn patient consent.

## Abbreviations

CA125: Cancer antigen 125
EOC: Epithelial ovarian cancer
FIGO: The international federation of gynecology and obstetrics
OS: Overall survival
PFS: Progression free survival
ROC: Receiver Operating Characteristic
